This article has been retracted.

# A Novel of New 7D Hyperchaotic System with Self-Excited Attractors and Its Hybrid Synchronization

**DOI:** 10.1155/2021/3081345

**Published:** 2021-12-30

**Authors:** Ahmed S. Al-Obeidi, Saad Fawzi Al-Azzawi, Abdulsattar Abdullah Hamad, M. Lellis Thivagar, Zelalem Meraf, Sultan Ahmad

**Affiliations:** ^1^Specialty of Mathematics, Gifted School of Nineveh, Directorate of Education, Mosul, Iraq; ^2^Department of Mathematics, College of Computer Science and Mathematics, University of Mosul, Mosul, Iraq; ^3^School of Mathematics, Madurai Kamaraj University, Madurai, Tamilnadu, India; ^4^Department of Statistics, Injibara University, Injibara, Ethiopia; ^5^Department of Computer Science, College of Computer Engineering and Sciences, Prince Sattam Bin Abdulaziz University, P.O.Box. 151, Alkharj 11942, Saudi Arabia

## Abstract

In this study, a novel 7D hyperchaotic model is constructed from the 6D Lorenz model via the nonlinear feedback control technique. The proposed model has an only unstable origin point. Thus, it is categorized as a model with self-excited attractors. And it has seven equations which include 19 terms, four of which are quadratic nonlinearities. Various important features of the novel model are analyzed, including equilibria points, stability, and Lyapunov exponents. The numerical simulation shows that the new class exhibits dynamical behaviors such as chaotic and hyperchaotic. This paper also presents the hybrid synchronization for a novel model via Lyapunov stability theory.

## 1. Introduction

In 1963, Lorenz introduces the first known system of the 3D chaotic model, which has just one positive Lyapunov exponent and two quadratic nonlinearities. Subsequently, Rössler introduced another 3D chaotic model in 1976 which also includes seven terms, with one quadratic nonlinearity. Several well-known paradigms of the 3D chaotic models are chaotic Chua's circuit, Liu model, and the Pan model [1–10].

In 1979, the first four-dimensional (4D) model with two positive Lyapunov exponents (LEs) including real variables is performed by Rössler, and various 4D hyperchaotic models have been discovered in the previous works. These models are distinguished to own two +ve LEs and the dimension of the hyperchaotic model is related to the number of +ve LEs so that the minimum dimension for the hyperchaotic model is four. To increase the number of +ve LEs, it the dimension of the model must be increased. Recently, there is great interest in construction of 5D models with three +ve LEs as the hyperchaotic Hu model 2009 [11, 12].

Due to its increased unpredictability and randomness, the chaotic model with a higher dimension is beneficial compared to the low dimension and has a superior performance compared to the standard 3D, 4D, and 5D models. To date, only a few studies on the subject have been increased, and many articles have been dedicated to the construction of new high-dimensional (6D) models with four +ve LEs [13, 14] and (7D) models with five +ve LEs [15, 16]

In 2018, Yang et al. construct a 6D model which contains 16 terms; three terms are nonlinearities and are described by [17]

(1) $$\begin{array}{c} \left\{\begin{array}{c} {\dot{x}}_{1}\left(t\right)=a\left(x_{2}-x_{1}\right)+x_{4}+rx_{6},\\ {\dot{x}}_{2}\left(t\right)=cx_{1}-x_{2}-x_{1}x_{3}+x_{5},\\ {\dot{x}}_{3}\left(t\right)=-bx_{3}+x_{1}x_{2},\\ {\dot{x}}_{4}\left(t\right)=dx_{4}-x_{1}x_{3},\\ {\dot{x}}_{5}\left(t\right)=-hx_{2}+x_{6},\\ {\dot{x}}_{6}\left(t\right)=k_{1}x_{1}+k_{2}x_{2}. \end{array}\right. \end{array}$$

The above system has four positive Lyapunov exponents:

(2) $$\begin{array}{c} \left\{\begin{array}{c} {\text{LE}}_{1}=0.4302,\\ {\text{LE}}_{2}=0.2185,\\ {\text{LE}}_{3}=0.1294,\\ {\text{LE}}_{4}=0.0775,\\ {\text{LE}}_{5}=-0.0001,\\ {\text{LE}}_{6}=-12.5222, \end{array}\right. \end{array}$$

where (*x*_1_(*t*), *x*_2_(*t*), *x*_3_(*t*), *x*_4_(*t*), *x*_5_(*t*), *x*_6_(*t*))^*T*^ ∈ *R*^6^ is the real state variables of the model (1), abdh ≠ 0, *a*, *b*, *c* are constant parameters, and *d*, *h*, *r*, *k*_1_, *k*_2_ are the control parameters.

To construct a hyperchaotic model, it is required to increase the dimension of a model. Based on state feedback control, we can add linear and nonlinear control (state variable) to the standard model [11–13].

The first pioneering study was introduced by Pecora and Carrol in 1990 for chaos synchronization of the abovementioned model which has received a lot of attention from many areas such as encryption [17], FPGA implementation [18], optimization [19–23], electronic circuits [24], and Engineering [25]. There have been various schemes for synchronization phenomena as complete synchronization [5, 7], antisynchronization [26], hybrid synchronization [27], projective synchronization [28], and generalized projective synchronization [3]. There are several reasons for this study. One is that a few works exist in the 7D model. The second reason led us to look for another method called the linear method. It is believed that the HS with another approach (linearization) can open the way for other kinds of synchronization phenomena.

## 2. The New 7D Hyperchaotic Model

A novel model of high-dimensional (7D) system presents via adding nonlinear controller *x*_7_; a 7D hyperchaotic model is constructed, which is described as

(3) $$\begin{array}{c} \left\{\begin{array}{c} {\dot{x}}_{1}\left(t\right)=a\left(x_{2}-x_{1}\right)+x_{4}+rx_{6}-x_{7},\\ {\dot{x}}_{2}\left(t\right)=cx_{1}-x_{2}-x_{1}x_{3}+x_{5},\\ {\dot{x}}_{3}\left(t\right)=-bx_{3}+x_{1}x_{2},\\ {\dot{x}}_{4}\left(t\right)=dx_{4}-x_{1}x_{3},\\ {\dot{x}}_{5}\left(t\right)=-hx_{2}+x_{6},\\ {\dot{x}}_{6}\left(t\right)=px_{1}+qx_{2},\\ {\dot{x}}_{7}\left(t\right)=x_{1}x_{2}-kx_{7}, \end{array}\right. \end{array}$$

where (*x*_1_(*t*), *x*_2_(*t*), *x*_3_(*t*), *x*_4_(*t*), *x*_5_(*t*), *x*_6_(*t*), *x*_7_(*t*))^*T*^ ∈ *R*^7^ is the real variables of (3), *a*, *b*, *c*, *d*, *h*, *r*, *k*_1_, *k*_2_ are the constant real parameters, and *k* is the parameter which determines the dynamical behavior. Fix *a*=10, *b*=8/3, *c*=28, *d*=2, *h*=9.9, *r*=1, *p*=1, *q*=2, and *k*=13.5; model (3) has a hyperchaotic attractor as explained in Figure 1. The new model includes 19 terms with four nonlinearities.

### 2.1. Equilibrium and Stability

Equal the right-hand side to zero, such that

(4) $$\begin{array}{c} \left\{\begin{array}{c} a\left(x_{2}-x_{1}\right)+x_{4}+rx_{6}-x_{7}=0,\\ cx_{1}-x_{2}-x_{1}x_{3}+x_{5}=0,\\ -bx_{3}+x_{1}x_{2}=0,\\ dx_{4}-x_{1}x_{3}=0,\\ -hx_{2}+x_{6}=0,\\ px_{1}+qx_{2}=0,\\ x_{1}x_{2}-kx_{7}=0. \end{array}\right. \end{array}$$

Solving system (4) leads to obtaining one origin point, and the Jacobian of (3) is

(5) $$\begin{array}{c} J\left(O\right)=\left[\begin{array}{ccccccc} -a & a & 0 & 1 & 0 & r & -1\\ c & -1 & 0 & 0 & 1 & 0 & 0\\ 0 & 0 & -b & 0 & 0 & 0 & 0\\ 0 & 0 & 0 & d & 0 & 0 & 0\\ 0 & -h & 0 & 0 & 0 & 1 & 0\\ p & q & 0 & 0 & 0 & 0 & 0\\ 0 & 0 & 0 & 0 & 0 & 0 & -k \end{array}\right]. \end{array}$$

The model is dissipative or nonconservative since sign of diverges is negative under the typical parameters; its divergent volume is given by

(6) $$\begin{array}{c} \text{div }V=\sum_{i=1}^{7}\frac{\partial {\dot{x}}_{i}}{\partial x_{i}}=-\left(a+1+b-d+k\right). \end{array}$$

Using |*J*(*O*) − *λI*|=0, *I*_7×7_ is the polynomial equation and roots at (*a*, *b*, *c*, *d*, *h*, *r*, *p*, *q*, *k*)=(10, 8/3, 28,2,9.9, 1,1,2,12), respectively,:

(7) $$\begin{array}{c} p\left(\lambda \right)=\lambda^{7}+\frac{71}{3}\lambda^{6}-\frac{1191}{10}\lambda^{5}-\frac{49529}{15}\lambda^{4}-\frac{1867}{2}\lambda^{3}+\frac{48935}{3}\lambda^{2}-\frac{13332}{5}\lambda +\frac{12768}{5},\\ \left\{\begin{array}{c} \lambda_{1}=2,\\ \lambda_{2}=-12,\\ \lambda_{3}=-\frac{8}{3},\\ \lambda_{4}=11.4755,\\ \lambda_{5}=-22.6229,\\ \lambda_{6,7}=0.0737\pm 0.3850i. \end{array}\right. \end{array}$$

It is clear that some roots are with positive real parts; therefore, the point *O* is unstable. Therefore, (3) has self-excited attractors (if the model possesses unstable equilibrium points, then it is called a system with self-excited attractors) [20, 29–35].

### 2.2. Analysis of Lyapunov Exponents

The simulation was implemented via Wolf Algorithm and MATLAB software 2020, with parameters *a*=10, *b*=8/3, *c*=28, *d*=2, *h*=9.9, *r*=1, *p*=1, *q*=2 and control parameter *k*=13.5, and the new model has five +ve Lyapunov spectra under initial conditions (0.1, 0.2, 0.3, 0.3, 0.2, 0.1, 0.4), and the corresponding five exponents are

(8) $$\begin{array}{c} \left\{\begin{array}{c} {\text{LE}}_{1}=0.4783,\\ {\text{LE}}_{2}=0.1688,\\ {\text{LE}}_{3}=0.0925,\\ {\text{LE}}_{4}=0.0501,\\ {\text{LE}}_{5}=0.0001,\\ {\text{LE}}_{6}=-12.3702,\\ {\text{LE}}_{7}=-13.5845, \end{array}\right.\\ \sum_{i=1}^{7}{\text{LE}}_{i}=-25.1647. \end{array}$$

Figure 2 displays these exponents with step=0.5 and tend=200. To show the effect of the control parameter *k* on the proposed model, fix *a*=10, *b*=8/3, *c*=28, *d*=2, *p*=1, *q*=2, *h*=9.9, *r*=1 and vary parameter *k*.  Table 1 demonstrates the new class changes into chaotic or hyperchaotic, and some corresponding parameters *k* are shown in Figure 3.

## 3. HS of the New 7D Hyperchaotic Model

Let us model (3) is the drive as

(9) $$\begin{array}{c} \left[\begin{array}{c} {\dot{x}}_{1}\\ {\dot{x}}_{2}\\ {\dot{x}}_{3}\\ {\dot{x}}_{4}\\ {\dot{x}}_{5}\\ {\dot{x}}_{6}\\ {\dot{x}}_{7} \end{array}\right]=\underset{A_{1}}{\underset{︸}{\left[\begin{array}{ccccccc} -a & a & 0 & 1 & 0 & r & -1\\ c & -1 & 0 & 0 & 1 & 0 & 0\\ 0 & 0 & -b & 0 & 0 & 0 & 0\\ 0 & 0 & 0 & d & 0 & 0 & 0\\ 0 & -h & 0 & 0 & 0 & 1 & 0\\ p & q & 0 & 0 & 0 & 0 & 0\\ 0 & 0 & 0 & 0 & 0 & 0 & -k \end{array}\right]}}\left[\begin{array}{c} x_{1}\\ x_{2}\\ x_{3}\\ x_{4}\\ x_{5}\\ x_{6}\\ x_{7} \end{array}\right]+\underset{B_{1}}{\underset{︸}{\left[\begin{array}{cccc} 0 & 0 & 0 & 0\\ 1 & 0 & 0 & 0\\ 0 & 1 & 0 & 0\\ 0 & 0 & 1 & 0\\ 0 & 0 & 0 & 0\\ 0 & 0 & 0 & 0\\ 0 & 0 & 0 & 1 \end{array}\right]}}\underset{C_{1}}{\underset{︸}{\left[\begin{array}{c} -x_{1}x_{3}\\ x_{1}x_{2}\\ -x_{1}x_{3}\\ x_{1}x_{2} \end{array}\right]}}, \end{array}$$

where *A*_1_, *B*_1_,  and *C*_1_ are the parameters and nonlinear part of (3), respectively. The response model is

(10) $$\begin{array}{c} \left[\begin{array}{c} {\dot{y}}_{1}\\ {\dot{y}}_{2}\\ {\dot{y}}_{3}\\ {\dot{y}}_{4}\\ {\dot{y}}_{5}\\ {\dot{y}}_{6}\\ {\dot{y}}_{7} \end{array}\right]=A_{2}\left[\begin{array}{c} y_{1}\\ y_{2}\\ y_{3}\\ y_{4}\\ y_{5}\\ y_{6}\\ y_{7} \end{array}\right]+\left(B_{2}C_{2}+\left[\begin{array}{c} u_{1}\\ u_{2}\\ u_{3}\\ u_{4}\\ u_{5}\\ u_{6}\\ u_{7} \end{array}\right]\right),C_{2}=\left[\begin{array}{c} -y_{1}y_{3}\\ y_{1}y_{2}\\ -y_{1}y_{3}\\ y_{1}y_{2} \end{array}\right], \end{array}$$

and let *U*=[*u*_1_, *u*_2_, *u*_3_, *u*_4_, *u*_5_, *u*_6_, *u*_7_]^*T*^ be the nonlinear controller to be constructed:

- If *A*_1_=*A*_2_ and *B*_1_=*B*_2_, then we refer to the identical model
- If *A*_1_ ≠ *A*_2_ or/and *B*_1_ ≠ *B*_2_, then refer to the nonidentical model (different)

The two models can be synchronized as *e*_*i*_=*y*_*i*_ − *αx*_*i*_, where

(11) $$\begin{array}{c} \alpha =\left\{\begin{array}{c} 1;\;i\;=1,3,5,7\left(\text{odd}\right),\\ -1;\;i=2,4,6\left(\text{even}\right), \end{array}\right. \end{array}$$

and satisfied that lim_*t*⟶*∞*_*e*_*i*_=0. Subtracting and adding of (10) from (9), we have the error dynamics as

(12) $$\begin{array}{c} {\dot{e}}_{1}=ae_{2}-2ax_{2}-ae_{1}+e_{4}-2x_{4}+re_{6}-2rx_{6}-e_{7}+u_{1},\\ {\dot{e}}_{2}=ce_{1}+2cx_{1}-e_{2}+e_{5}+2x_{5}-y_{1}e_{3}+x_{3}e_{1}-2y_{1}x_{3}+u_{2},\\ {\dot{e}}_{3}=-be_{3}+e_{1}e_{2}-x_{2}e_{1}+x_{1}e_{2}-2x_{1}x_{2}+u_{3},\\ {\dot{e}}_{4}=de_{4}-y_{1}e_{3}+x_{3}e_{1}-2y_{1}x_{3}+u_{4},\\ {\dot{e}}_{5}=-he_{2}+2hx_{2}+e_{6}-2x_{6}+u_{5},\\ {\dot{e}}_{6}=pe_{1}+2px_{1}+qe_{2}+u_{6},\\ {\dot{e}}_{7}=-ke_{7}+e_{1}e_{2}-x_{2}e_{1}+x_{1}e_{2}-2x_{1}x_{2}+u_{7}. \end{array}$$

**Theorem 1 .**

Models (9) and (10) are globally and asymptotically HS via the nonlinear control *U* of equation (12) which is designed as follows:

(13) $$\begin{array}{c} \left\{\begin{array}{c} u_{1}=2ax_{2}+2x_{4}-re_{6}+2rx_{6}-ce_{2}-x_{3}e_{2}-pe_{6},\\ u_{2}=-ae_{1}-2cx_{1}-2x_{5}+2y_{1}x_{3}-x_{1}e_{3}-qe_{6}-x_{1}e_{7},\\ u_{3}=y_{1}e_{2}-e_{1}e_{2}+x_{2}e_{1}+2x_{1}x_{2}+y_{1}e_{4},\\ u_{4}=-2\text{d}e_{4}-e_{1}-x_{3}e_{1}+2y_{1}x_{3},\\ u_{5}=-2hx_{2}+2x_{6}-e_{5},\\ u_{6}=-2px_{1}-e_{5}-e_{6},\\ u_{7}=e_{1}-e_{1}e_{2}+x_{2}e_{1}+2x_{1}x_{2}. \end{array}\right. \end{array}$$

**Proof**

Inserting the above control in (12), we obtain

(14) $$\begin{array}{c} \left\{\begin{array}{c} {\dot{e}}_{1}=ae_{2}-ae_{1}+e_{4}-e_{7}-ce_{2}-x_{3}e_{2}-pe_{6},\\ {\dot{e}}_{2}=ce_{1}-e_{2}+e_{5}-y_{1}e_{3}+x_{3}e_{1}-ae_{1}-x_{1}e_{3}-qe_{6}-x_{1}e_{7},\\ {\dot{e}}_{3}=-be_{3}+x_{1}e_{2}+y_{1}e_{2}+y_{1}e_{4},\\ {\dot{e}}_{4}=-\text{d}e_{4}-y_{1}e_{3}-e_{1},\\ {\dot{e}}_{5}=-he_{2}+e_{6}-e_{5},\\ {\dot{e}}_{6}=pe_{1}+qe_{2}-e_{5}-e_{6},\\ {\dot{e}}_{7}=-ke_{7}+x_{1}e_{2}+e_{1}. \end{array}\right. \end{array}$$

The characteristic equation and roots are as

(15) $$\begin{array}{c} \lambda^{7}+\frac{89}{3}\lambda^{6}+\frac{6529}{10}\lambda^{5}+\frac{238931}{30}\lambda^{4}-\frac{1182143}{30}\lambda^{3}+\frac{291515}{3}\lambda^{2}+\frac{1944721}{15}\lambda +\frac{1163288}{15}=0,\\ \left\{\begin{array}{c} \lambda_{1}=-\frac{8}{3},\\ \lambda_{2}=-11.9657,\\ \lambda_{3}=-2.0021,\\ \lambda_{4,5}=-1.1984\pm 1.4399i,\\ \lambda_{6,7}=-5.3177\pm 17.8223i. \end{array}\right. \end{array}$$

Clearly, all roots are with negative real parts; the linearization approach achieved the HS between (9) and (10).

Now, in second approach, we construct the auxiliary (Lyapunov) function as *V*(*e*_*i*_)=*e*^*T*^*Pe*, i.e.,

(16) $$\begin{array}{c} V\left(e_{i}\right)={\left[e_{1},e_{2},e_{3},e_{4},e_{5},e_{6},e_{7}\right]}^{T}\underset{P}{\underset{︸}{\left[\begin{array}{ccccccc} 0.5 & 0 & 0 & 0 & 0 & 0 & 0\\ 0 & 0.5 & 0 & 0 & 0 & 0 & 0\\ 0 & 0 & 0.5 & 0 & 0 & 0 & 0\\ 0 & 0 & 0 & 0.5 & 0 & 0 & 0\\ 0 & 0 & 0 & 0 & 5/99 & 0 & 0\\ 0 & 0 & 0 & 0 & 0 & 0.5 & 0\\ 0 & 0 & 0 & 0 & 0 & 0 & 0.5 \end{array}\right]}}\left[\begin{array}{c} e_{1}\\ e_{2}\\ e_{3}\\ e_{4}\\ e_{5}\\ e_{6}\\ e_{7} \end{array}\right]. \end{array}$$

The derivative of the above function *V*(*e*_*i*_) is

(17) $$\begin{array}{c} \dot{V}\left(e_{i}\right)=e_{1}{\dot{e}}_{1}+e_{2}{\dot{e}}_{2}+e_{3}{\dot{e}}_{3}+e_{4}{\dot{e}}_{4}+\frac{10}{99}e_{5}{\dot{e}}_{5}+e_{6}{\dot{e}}_{6}+e_{7}{\dot{e}}_{7},\\ \dot{V}\left(e\right)=e_{1}\left(ae_{2}-ae_{1}+e_{4}-e_{7}-ce_{2}-x_{3}e_{2}-pe_{6}\right)+e_{2}\left(ce_{1}-e_{2}+e_{5}-y_{1}e_{3}+x_{3}e_{1}-ae_{1}-x_{1}e_{3}-qe_{6}-x_{1}e_{7}\right)\\ +e_{3}\left(-be_{3}+x_{1}e_{2}+y_{1}e_{2}+y_{1}e_{4}\right)+e_{4}\left(\;-de_{4}-y_{1}e_{3}-e_{1}\right)+\frac{10}{99}e_{5}\left(-he_{2}+e_{6}-e_{5}\right)+e_{6}\left(pe_{1}+qe_{2}-e_{5}-e_{6}\right)+e_{7}\left(-ke_{7}+x_{1}e_{2}+e_{1}\right),\\ \dot{V}\left(e_{i}\right)=-{\left[e_{1},e_{2},e_{3},e_{4},e_{5},e_{6},e_{7}\right]}^{T}\underset{Q}{\underset{︸}{\left[\begin{array}{ccccccc} 10 & 0 & 0 & 0 & 0 & 0 & 0\\ 0 & 1 & 0 & 0 & 0 & 0 & 0\\ 0 & 0 & 8/3 & 0 & 0 & 0 & 0\\ 0 & 0 & 0 & 2 & 0 & 0 & 0\\ 0 & 0 & 0 & 0 & 10/99 & 0 & 0\\ 0 & 0 & 0 & 0 & 0 & 1 & 0\\ 0 & 0 & 0 & 0 & 0 & 0 & 12 \end{array}\right]}}\left[\begin{array}{c} e_{1}\\ e_{2}\\ e_{3}\\ e_{4}\\ e_{5}\\ e_{6}\\ e_{7} \end{array}\right], \end{array}$$

where *Q*=diag(10,1, 8/3, 2, 10/99, 1,12), so *Q* > 0. Consequently, $\dot{V}\left(e_{i}\right)<0$ on *R*^7^. The nonlinear controller realized the HS between models (9) and (10).

For simulation results, the initial values are (15,2,0, −2, −3,0) and (−15, −10, −8,6,0, −4) to illustrate the HS that happened between (9) and (10) numerically. Figures 4 and 5 check these results numerically, respectively.

## 4. Conclusions

In this paper, a novel class 7D model with a self-excited attractor and multiple positive Lyapunov exponents has been proposed via a state feedback controller. Furthermore, some features of dynamical behaviors such as equilibria points, stability, and Lyapunov exponents are investigated, as well as hybrid synchronization between two new identical models, are rigorously derived and studied by designing a suitable controller, based on nonlinear control strategy with two analytical methods: Lyapunov's and linearization approach. The new system may have a good application in the field of encryption and nonlinear circuits.

## Figures and Tables

**Figure 1:** The attractors of new model: (a) *x*_2_ − *x*_6_ − *x*_7_ space, (b) *x*_7_ − *x*_2_ plane, (c) *x*_4_ − *x*_7_ plane, and (d) *x*_4_ − *x*_6_ plane.

**Figure 2:** Lyapunov spectrum of the new 7D model.

**Figure 3:** Typical dynamical behaviors of (3) at different control parameters *k*. (a) *k* = 0.5. (b) *k* = 0.5. (c) *k* = 0.8. (d) *k* = 0.8. (e) *k* = 4.25. (f) *k* = 4.25.

**Figure 4:** HS between models (9) and (10) with nonlinear control (13).

**Figure 5:** The convergence of models (12) with nonlinear controllers (13).

**Table 1:** Dynamics of (3) versus control parameter *k*.

*k*	LE_1_	LE_2_	LE_3_	LE_4_	LE_5_	LE_6 _	LE_7_	Signs of LE

0.18	0.0306	0.0060	−0.1588	−0.3153	−1.3681	−2.1789	−7.8652	(+, ≈0, −, −, −, −, −)
0.55	0.4753	0.1636	0.0082	−0.0094	−0.5403	−1.6395	−10.6733	(+, +, ≈0, ≈0, −, −, −)
0.74	0.6136	0.1414	−0.0008	−0.0584	−0.7603	−1.3147	−11.026	(+, +, 0, −, −, −, −)
0.85	0.4863	0.0857	−0.032	−0.0005	−0.8137	−1.2039	−11.1011	(+, +, +, 0, −, −, −)
0.88	0.5951	0.1517	−0.0008	−0.0402	−0.8021	−1.3026	−11.146	(+, +, 0, −, −, −, −)
1.01	0.5266	0.9952	00388	0.0001	−0.8955	−1.171	−11.2735	(+, +, +, 0, −, −, −)
12.99	0.3734	0.1941	0.1386	0.0470	−0.0005	−12.1641	−13.2435	(+, +, +, +, 0, −, −)
13.5	0.4783	0.1688	0.0925	0.05011	0.0001	−12.3701	−13.5845	(+, +, +, +, 0, −, −)

## Data Availability

The data underlying the results presented in the study are available within the article.
